# Exogenous H_2_S Protects against Septic Cardiomyopathy by Inhibiting Autophagy through the AMPK/mTOR Pathway

**DOI:** 10.1155/2022/8464082

**Published:** 2022-06-10

**Authors:** YuHan Zhao, QingHong Cheng

**Affiliations:** ^1^Shihezi University School of Medicine, Shihezi 832000, China; ^2^The First Affiliated Hospital of Shihezi University, Shihezi 832000, China

## Abstract

**Background:**

Given the cardioprotective role of autophagy, this study aimed to investigate the protective effect of exogenous H_2_S (NaHS) on infectious cardiomyopathy through the inhibition of the AMPK/mTOR pathway.

**Methods:**

In this study, sepsis models were established by cecal ligation and puncture (CLP) induction in vivo and intraperitoneal injection of NaHS was performed. Autophagy- and apoptosis-related proteins were observed by western blot, isolated myocardial tissue morphology was observed by hematoxylin-eosin (H&E) staining, and myocardial apoptosis was evaluated by the tunnel method. The ultrastructure of autophagy was observed by using an electron transmission electron microscope.

**Results:**

In an SD rat model of cecum ligation puncture-induced sepsis, the level of autophagy-related proteins was significantly increased, and hematoxylin and eosin staining showed irregular myocardial bands and swollen cardiomyocytes. Following NaHS treatment, the level of autophagy-related proteins decreased, and electron transmission microscopy revealed decreased autophagosomes. Echocardiography suggested an increase in ejection fraction and significant relief of myocardial inhibition.

**Conclusions:**

Our results suggest that NaHS treatment can attenuate the cellular damage caused by excessive autophagy through the AMPK/mTOR pathway.

## 1. Introduction

According to Rudd and Johnson, while age-standardized sepsis has declined, sepsis remains one of the highest causes of death worldwide [1]. Sepsis is a systemic inflammatory response caused by infection, which rapidly involves multiple vital organs. The cardiac dysfunction caused by such inflammation is termed septic cardiomyopathy, which is associated with increased sepsis-associated mortality [2]. The pathogenesis of septic cardiomyopathy is highly complex and diverse. The studies by Galley and Joshi et al. demonstrated that cardiac dysfunction in sepsis is associated with mitochondrial dysfunction and a calmodulin imbalance [3, 4]. Recently, the role of autophagy in cardiac dysfunction during sepsis has received wide attention. Autophagy is a highly conserved cellular degradation process that is vital for maintaining the cellular stress response and steady-state conditions [5, 6]. Moreover, autophagy is involved in the maintenance of the stability of the normal intracellular environment by eliminating damaged proteins, abnormal protein aggregates, and damaged organelles [7, 8]. Moreover, autophagy is adaptive as it remains relatively stable during normal physiological activities to maintain the survival of the organism; however, under conditions of severe stress, both excessive and inadequate autophagy may lead to massive self-degradation of cellular contents or an accumulation of toxic substances as both outcomes eventually lead to cell death [9]. As shown by Tuerdi et al., increased autophagic flow protects the myocardium against sepsis in cardiac dysfunction. Since beclin-1-dependent autophagy can improve cardiac function and reduce inflammation and fibrosis, thereby playing a cardioprotective role [10, 11]. It has also been shown that autophagy instantaneously increases at the beginning of sepsis injury and subsequently decreases over time [12]; thus, it has been concluded that adjusting the autophagic flux at the appropriate time points is beneficial for improving sepsis-induced myocardial injury. Hydrogen sulfide (H_2_S) was previously considered to be a typical toxic gas; however, in recent years, it has been considered to be a third gas conductor in addition to nitric oxide (NO) and carbon monoxide (CO) [13]. In the study by Chen et al., NaSH was found to increase the level of endogenous H_2_S, which inhibited excessive autophagy induced by the ROS-AMPK pathway [15]. H_2_S can easily cross cellular membranes because it is five times more soluble in cell membranes than in water, and it is involved in a wide range of signaling related to inflammation and autophagy [14]. Another H_2_S donor, GYY4137, was found to inhibit the expression of inducible nitric oxide synthase (iNOS) and NO production in endotoxemic lungs, suggesting that GYY4137 may be involved in antioxidant, anti-nitrification, and anti-inflammatory responses [16]. In the study by Nie et al., it was demonstrated that H_2_S can ameliorate myocardial fibrosis in mice with alcoholic cardiomyopathy by downregulating autophagy through the PI3K/AKT signaling pathway [17].

In summary, multiple exogenous H_2_S donors have been shown to modulate autophagy and counteract inflammation and oxidative stress through multiple signaling pathways as well as attenuate septic organ damage [18, 19]. In septic cardiomyopathy, the relationship between H_2_S and autophagy has not been fully elucidated; therefore, in vivo studies were used in this study to identify potential mechanisms of autophagy and exogenous H_2_S (NaHS) donors for the treatment of sepsis.

## 2. Materials and Methods

Animal experimental procedures were performed in accordance with the regulations of the Animal Protection Committee of Shihezi University, and all experimental protocols were approved by the Animal Protection and Use Committee of Shihezi University. A total of 80 adult male Sprague–Dawley rats (7-8 weeks old; weight 227.14 g ± 10.36 g) were purchased from the Animal Center of Xinjiang Medical University, China, and housed at the Animal Science Center of the Shihezi University School of Medicine under room temperature (20°C–22°C) [1], humidity (50%–60%), and normal air conditions (12 h light-dark cycle).

### 2.1. Establishment of a Sepsis Model

Rats were anesthetized by an intraperitoneal injection of 40 mg/kg pentobarbital, a median incision of 1.5 cm was made, and the cecum was identified and gently removed. The cecum was ligated with a thin wire and punctured with an 18-gauge needle at several different locations in the cecum to induce sepsis. The cecum was then returned to the abdominal cavity and the abdominal wall and skin were closed. Antibiotics and fluid resuscitation were not used during the study. Rats were randomly divided into seven groups: (1) sham; (2) CLP; (3) NaHS treatment; (4) CLP NaHS treatment; (5) endogenous hydrogen sulfide inhibitor (PAG) treatment; (6) CLP PAG treatment; (7) CLP, NaHS, and PAG treatment groups. Exogenous hydrogen sulfide donor (NaHS) was injected intraperitoneally. Rats were intraperitoneally injected with NaHS (8.9 *μ*mol/kg). All doses selected for PAG (50 mg/kg) were based on the results of our previous study [20]. The control group was administered the same amount of normal saline and all rats were killed 6 h after the induction of sepsis. Heart tissues were immediately removed after death. Each heart tissue specimen was fixed in paraformaldehyde (4%) for histomorphometric analysis and the remaining tissue was stored at −80°C for use in other experiments.

### 2.2. Hematoxylin-Eosin (HE) Staining

The rat myocardial tissue was removed and fixed overnight in 4% paraformaldehyde, embedded in paraffin, stained with hematoxylin for 5 min, rinsed with running water for 30 s, stained with 5% eosin for 3 min, rinsed for 30 s, mounted, and observed under a microscope.

### 2.3. Myocardial Enzyme Assay

Creatine kinase isoenzyme CKMB and lactate dehydrogenase LDH were detected with an automatic biochemical analyzer (Modular DPP H7600; Roche Diagnostics, Basel, Switzerland).

### 2.4. Echocardiogram

The rats were anesthetized with pentobarbital 6 h after CLP. Echocardiography was measured by using an M-mode echocardiography system with a 10 MHz linear transducer. Left ventricular ejection fraction (LVEF) and left ventricular fractional shortening (LVFS) were analyzed by using computer algorithms.

### 2.5. Transmission Electron Microscopy

Myocardial tissue from the rats was cut into 2-mm cubes and fixed with 2.5% glutaraldehyde. After dehydration by rising in an ethanol series and embedding in epoxy resin, ultrathin sections were cut and stained with uranyl acetate and lead citrate. All ultrastructural analyses were performed blindly and without bias, using micrographs taken with a Philips CM120 electron microscope.

### 2.6. Immunofluorescence

The cells were washed with ice-cold PBS, and 4% paraformaldehyde was fixed for 15 min at room temperature. Next, the cells were permeabilized with 0.2% Triton X-100. The cells were incubated with anti-LC3-II (1 : 100, Abcam) for 2 h at room temperature. The cells were washed three times with cold PBS and incubated with an anti-rabbit secondary antibody (1 : 800) (Invitrogen, USA) for 1 h at room temperature. The cell nuclei were stained with 4′,6-diamidino-2-phenylindole (DAPI) (Sigma-Aldrich) and observed by fluorescence microscopy (OLYMPUS-IX73P2F).

### 2.7. Western Blot

The total protein was extracted with cell lysis buffer (Solarbio cat#R0010) followed by the addition of protease and phosphorylated protease inhibitors. The protein concentration was determined using a spectrophotometer (Thermo Fisher). Next, 10 *μ*L of total protein was loaded onto 6%–12% SDS-PAGE gels and transferred to PVDF membranes. The membranes were incubated with primary and secondary antibodies. Protein signals were detected using the ECL method. Primary antibodies used in this study included anti-p-AMPK (1 : 1000, Abcam32047), anti- AMPK (1 : 1000, Abcam133448), anti-p62 (1 : 1000, Ab109012), anti-beclin-1 (1 : 1000, Ab210498), anti-mTOR (1 : 1000, Abcam134903), anti-p-mTOR (1 : 1000, Abcam109268), anti-caspase-3 (1 : 1000, Ab13847), anti-caspase-9 (1 : 1000, Ab184786), and anti-LC3-II (1 : 1000, Ab192890). All primary antibodies were incubated overnight at 4°C. The HRP-labeled goat anti-rabbit lgG H&L (1 : 10,000) was incubated for 2 h at room temperature.

### 2.8. Assessment of Apoptosis

Apoptotic myocardial tissue was stained for apoptosis using the TDT-mediated dUTP end-labeling (TUNEL) method according to the manufacturer's instructions associated with an in situ cell death detection kit (Roche, Mannheim, Germany). After fixing the tissue sections or cell cultures with 4% paraformaldehyde for 15 min at room temperature, the cells were permeabilized with 0.2% Triton X-100 for 15 min at room temperature. The reaction mixture was incubated with the TUNEL fraction for 60 min at 37°C. The samples were subsequently immersed in DAPI, and the nuclei were examined. Finally, the nuclei were rinsed three times with PBS, observed under a laser confocal scanning microscope and photographed.

## 3. Results

### 3.1. Sepsis Causes Impaired Cardiac Function in Rats

H&E staining of the heart sections following CLP treatment revealed blurred or absent transverse myocardial lines in the cardiomyocytes of the CLP rats, a sign of myocardial injury. H_2_S treatment improved the cardiomyocyte morphology in rats. In contrast, the cardiomyocyte injury was more severe in the group treated with the H_2_S inhibitor, PAG. The cells were loosely arranged and disorganized (Figure 1). The cardiac function of the rats was measured by echocardiography. At 6 h after CLP, the myocardial volume at the end-diastole and end-systole was significantly increased in the CLP rats (Figures 1(b) and 1(e)), whereas the overall left ejection fraction was reduced. The levels of serum CKMB and LDH were increased in the CLP group. Compared with the Sham rats, H_2_S significantly reduced the production of these injurious substances. While PAG inhibited the effect of endogenous H_2_S, the levels of serum CKMB and LDH were significantly higher in the PAG-treated CLP rats compared to that in the CLP group (Figures 1(c) and 1(d)).

### 3.2. Overautophagy Causes Impaired Cardiac Function in Septic Rats

To determine the effect of H_2_S on the regulation of the AMPK/mTOR pathway and thus cardiac protection, we determined the expression of the related proteins by western blot. We determined the upstream proteins p-AMPK, AMPK, p-mTOR, and mTOR. p-AMPK was activated with elevated expression in the CLP group, while the opposite was true for p-mTOR (Figures 2(d) and 2(e)). Activation of p-AMPK leads to activation of the downstream autophagy-related proteins (e.g., LC3 and p62). LC3 is now one of the most recognizable markers of autophagy, and an increased LC3-II is an indicator of autophagy. Moreover, reduced expression of the ubiquitin-binding protein, p62, is characterized by the activation of autophagy [21]. H_2_S was found to reduce autophagy flux in CLP rats compared to sham-operated rats, and the opposite trend was observed in PAG-treated CLP rats (Figure 2(a)). The results suggest that the LC3-II was higher in the CLP rats than in the sham rats, and the LC3-II was higher in PAG-treated CLP rats than in the CLP mice (Figure 2(h)). p62 expression was reduced in the PAG-treated CLP group compared with the CLP group and was lower than that in the sham group (Figure 2(g)). We also examined the apoptosis-related proteins, c-caspase3, and c-caspase9. Interestingly, autophagy was activated in the CLP group, as well as in the PAG-treated CLP group, while the apoptosis-related proteins were similarly elevated (Figures 2(i) and 2(j)). Furthermore, the number of autophagosomes was observed by transmission electron microscopy. The data showed an increase in the number of autophagosomes in the CLP group compared to the sham group (Figures 2(b) and 2(k)). In addition, tunnel fluorescence imaging showed increased apoptosis in the cardiomyocytes of the CLP rats compared to the sham group. H_2_S treatment reduced the occurrence of apoptosis, whereas PAG treatment exacerbated apoptotic expression (Figures 2(c) and 2(l)).

## 4. Discussion

The inhibition of myocardial function is one of the distinguishing features of septic cardiomyopathy [22]. Since the restoration of cardiac function is essential for improving survival in septic patients [23], there is an urgent need to understand the pathogenesis of sepsis. The results of our study revealed that (1) sepsis inhibits myocardial function; (2) autophagic flux increases as a compensatory mechanism in early sepsis; (3) excessive levels of autophagy exacerbate myocardial dysfunction; and (4) NaHS reduces autophagic flux and protects cardiomyocytes. The primary manifestations of septic cardiomyopathy are systolic dysfunction and a reduced ejection fraction [24]. The echocardiography revealed a decrease in the left ventricular shortening fraction (LVFS) and left ventricular ejection fraction (LVEF) in the CLP rats (Figures 1(e) and 1(f)), along with an increase in LDH and CKMB levels (Figures 1(c) and 1(d)).

An increasing number of studies have shown that autophagic activity is elevated during the hyperdynamic phase of sepsis and decreased in the late phase [25, 26]. AMP-activated protein kinase (AMPK) activates the autophagic pathway and plays a key role in the maintenance of cellular energy. In contrast, the mammalian target of rapamycin (mTOR) is an established inhibitor of autophagy [27].26. Autophagy is a process by which cells degrade and recycle themselves. There are three main stages, which begin with the formation of autophagic vacuoles, followed by the transport of cargo (unfolded proteins or damaged organelles) into the double-membrane structure of the autophagosome, and finally binding to lysosomes, where the contents are degraded [28]. The western blot results in this study showed that p-AMPK activation was accompanied by p-mTOR downregulation (Figures 2(d) and 2(e)), indicating activation of the AMPK/mTOR pathway, followed by the detection of the downstream autophagy signature protein LC-3-II, in our experiments. LC3-II levels were significantly higher in the sepsis group, suggesting that the levels of autophagy were significantly increased in the early stages of sepsis, as also confirmed in the study by Takahashi et al. Conditions of either excessive or insufficient autophagy will lead to cell death. In a study by Yutaka et al., it was found that the downregulation of autophagy via the inhibition of beclin-1 was protective during Ischemia-reperfusion (I/R) model in rats, and a knockdown of beclin-1 inhibition in autophagy also increased the viability of cultured cardiomyocytes in vitro [29]. Moreover, a study by Jiang et al. demonstrated that blocking the AMPK-ULK1 pathway can ameliorate BCAA-induced excessive autophagy mediated by myocardial injury. The western blot revealed an increased level of autophagy and apoptotic proteins in the CLP group. We also observed the number of autophagosomes by transmission electron microscopy and found that the number of autophagosomes in the myocardium of CLP rats was significantly increased. In contrast, a small number of autophagy-lysosomes was observed, and TUNEL fluorescence also indicated that apoptosis was significantly increased in the CLP group. The above results confirm our speculation that a high level of autophagy in early septic cardiomyopathy may be detrimental. Activation of the caspase family is an indispensable marker of apoptosis [30]. Autophagic cell death (PCD-2A) is the second mode of programmed cell death that differs from apoptosis that has recently been identified [31, 32], and beclin-1/bcl-2 represents the autophagy-apoptosis pathway. The point of CHOP crosstalk has been found to induce the nuclear translocation of Bcl-2 to release beclin-1 and induce autophagic apoptosis in hepatocellular carcinoma cells [33]. Moreover, the downregulation of Bcl-2 has been shown to increase autophagic apoptosis in human leukemia cells [34]. Bcl-2 also inhibits beclin-1-mediated autophagy under conditions of starvation [35]. In our study, experiments revealed that beclin-1 was upregulated in the sepsis group (Figures 2(a) and 2(f)). Based on the above evidence, we hypothesize that a beclin-1-dependent autophagic apoptotic pathway may also be activated in septic rats. Moreover, since single time points during autophagosome formation can be used to assess the extent of autophagy [36], we evaluated the extent of autophagy based on the number of autophagosomes and the level of autophagy-related proteins in a 6 h model of sepsis in rats. Although we observed several autophagosomes in the CLP group of rats under electron microscopy, autophagy-associated lysosomes were rarely observed (Figure 2(b)). Perhaps this excess of ineffective “autophagosomes” did not serve to remove harmful substances but rather activated the relevant apoptotic pathways.

H_2_S is a biologically active gas signaling molecule that plays a regulatory role in various physiological pathways [37]. The cardioprotective effects of H_2_S are well known [38–40], and the dual role of autophagy in the cardiovascular system remains a controversial topic. To maintain cardiovascular homeostasis, the maintenance of appropriate levels of autophagy is critical. H_2_S acts as a transducer in autophagy, which both up- and downregulates autophagy and plays a role in pathological processes in different tissues, although NaHS improves myocardial suppression in sepsis. However, it appears that the effect is not obvious in normal myocardial tissue, as the addition of NaHS to the normal groups was not associated with significant alteration in the levels of autophagy and apoptosis-related proteins in experiments. In our study, we observed that the administration of NaSH, attenuated myocardial depression in septic rats, and echocardiography revealed an increased ejection fraction and reduced heart rate. In addition, the administration of PAG, an endogenous H_2_S inhibitor, to CLP rats showed a further increase in the level of LDH and CKMB, which was possibly due to the inhibition of endogenous H_2_S activity by PAG, and resulted in the failure to exert myocardial protection. HE staining further confirmed this hypothesis, and western blot results showed that the administration of NaHS resulted in decreased levels of autophagy. The western blot results revealed decreased levels of autophagy, apoptosis-related proteins (Figure 2(a)), and the fluorescence intensity in the TUNEL staining of apoptotic cells (Figure 2(c)). Given the addition of NaHS, there was a decrease in autophagic vesicles and increased autolysosomes visible under transmission electron microscopy in the CLP rat group, Taken together, we conclude that excessive autophagy induced by AMPK/mTOR in sepsis leads to myocardial dysfunction. In addition, H_2_S, a novel gas signaling molecule, can attenuate this excessive autophagy and exert a protective effect on the myocardium. Thus, the findings of this study may provide a novel therapeutic strategy for the treatment of septic cardiomyopathy.

## Figures and Tables

**Figure 1:** Sepsis causes impaired cardiac function in rats. (a) Histopathological changes in the cardiac muscle. (b) Representative images of M-mode echocardiograms (*n* = 4); (c) CKMB (d) LDH (e) LVEF (f) LVFS; Scale bar = 100 *μ*m. Data were expressed as mean ± SEM. ^*∗*^*P* < 0.05 vs. sham group; ^*#*^*P* < 0.05 vs. CLP group. All the experiments were repeated three times.

**Figure 2:** Exogenous H2S inhibits excessive autophagy to reduce myocardial injury. (a) The expression of autophagy-related protein by Western blot analysis. (b) Representative images of myocardial autophagosome ultrastructural morphology underwent different treatments. Scale bar. = 5 *μ*m, 1 *μ*m (c) Representative TUNEL staining images; Scale bar = 50 *μ*m ((d)–(j)). The quantitative analysis of p-AMPK, p-mtor, beclin-1, p62, LC3-II, cleaved-caspase-3 and cleaved-caspase-9 by image J. (k) The number of autophagosomes in different treatment groups. All data are expressed as the mean ± SD. (l) Percentage of TUNEL-positive nuclei. ^*∗*^*P* < 0.05 vs. sham group; ^*#*^*P* < 0.05 vs. CLP group. All the experiments were repeated three times.

## Data Availability

No data were used to support this study.
